RETRACTED

# Pediatric Acute Dacryocystitis and Orbital Cellulitis With Concurrent COVID-19 Infection: A Case Report

**DOI:** 10.7759/cureus.46559

**Published:** 2023-10-05

**Authors:** Saleh Ghulaysi, Fatima Alhumaid, Manar Almania, Nouf AlQurashi, Ahmed Abdelaziz

**Affiliations:** 1 General Practice, Jazan University, Jazan, SAU; 2 General Practice, Imam Abdulrahman Bin Faisal University, Dammam, SAU; 3 General Practice, Majmaah University, Al-Majma'ah, SAU; 4 General Practice, King Saud bin Abdulaziz University for Health Sciences, Riyadh, SAU; 5 Ophthalmology, Dallah Hospital, Riyadh, SAU

**Keywords:** case report, computed tomography, covid-19, subperiosteal abscess, orbital cellulitis, acute dacryocystitis

## Abstract

Acute dacryocystitis and orbital cellulitis are conditions with serious implications, particularly among pediatric patients. The co-occurrence of these conditions in children is rare, and their association with coronavirus disease 2019 (COVID-19) infection introduces a unique dimension. We present the case of a five-year-old boy who presented to the pediatric emergency department with left periorbital swelling, erythema, and excessive tearing. He had a history of low-grade fever and rhinorrhea, raising concerns about COVID-19. Upon physical examination, we observed significant periorbital swelling and erythema, accompanied by conjunctival injection and chemosis. The diagnosis encompassed acute dacryocystitis and cellulitis, with subsequent confirmation of COVID-19 through testing. Imaging confirmed the presence of post-septal cellulitis and ethmoid sinus opacification. The patient received intravenous antibiotics, leading to clinical improvement and eventual discharge for outpatient follow-up. This case underscores the importance of maintaining a high index of suspicion for unusual presentations in pediatric patients. Successful management involved a multidisciplinary approach, emphasizing the significance of promptly initiating antibiotic therapy and adopting conservative measures for nasolacrimal duct obstruction.

## Introduction

Acute dacryocystitis is a relatively uncommon but potentially serious ophthalmic condition, especially in the pediatric population. Dacryocystitis is an infection of the lacrimal sac and nasolacrimal duct, typically presenting with periorbital erythema, swelling, and excessive tearing. Orbital cellulitis, on the other hand, refers to an infectious process involving the soft tissues surrounding the eye, which can lead to severe complications if not promptly diagnosed and treated [1]. The coexistence of acute dacryocystitis and orbital cellulitis in a pediatric patient is relatively rare, and its association with coronavirus disease 2019 (COVID-19) infection adds a unique dimension to this clinical scenario.

RETRACTED

The COVID-19 pandemic has brought to light various atypical manifestations of the disease, affecting not only the respiratory system but also other organ systems [2]. While ocular symptoms of COVID-19 are well documented, their association with orbital infections remains a subject of ongoing research [1]. This case report highlights the importance of considering uncommon orbital infections in pediatric patients, even in the presence of mild respiratory symptoms or asymptomatic COVID-19 infection.

## Case presentation

A five-year-old male child presented to our pediatric emergency department with a chief complaint of left periorbital swelling, erythema, and excessive tearing that had been progressively worsening over the past 72 hours. The child's parents reported that he had experienced low-grade fever (maximum recorded temperature 100.5°F) and rhinorrhea for the past week, which had prompted them to seek medical evaluation for potential COVID-19 infection. Apart from this, the child's past medical history was unremarkable, with no prior ocular or systemic illnesses.

On physical examination, the patient appeared ill but was conscious and oriented. Notably, there was marked erythema and edema of the left upper and lower eyelids. The periorbital swelling extended to the medial canthus, with tenderness to palpation. The left eye exhibited marked conjunctival injection, chemosis, and excessive tearing, obscuring the visualization of the globe. Ocular motility was intact, and no proptosis or changes in visual acuity were noted. There was no purulent discharge from the eye, but the lacrimal sac area appeared tense upon palpation.

Given the clinical presentation, we were concerned about the possibility of acute dacryocystitis and cellulitis. Given the ongoing COVID-19 pandemic, a nasopharyngeal swab was obtained for SARS-CoV-2 reverse transcription-polymerase chain reaction testing, which subsequently returned positive.

Laboratory investigations revealed elevated inflammatory markers, including a white blood cell count of 14,200/mm^3^ (normal range: 4,500-11,000/mm^3^) with a predominance of neutrophils, and an elevated C-reactive protein level of 17.8 mg/dL (normal range: <0.5 mg/dL). Blood cultures were obtained and showed no growth of microorganisms.

A contrast-enhanced computed tomography (CT) scan of the orbits and paranasal sinuses was performed, revealing diffuse soft-tissue swelling in the pre-septal and post-septal regions of the left orbit, indicative of pre-septal and post-septal cellulitis. Additionally, the CT scan showed subperiosteal cellulitis involving the left orbit and complete opacification of the ethmoid sinus, confirming the diagnosis of orbital cellulitis (Figure 1).

RETRACTED

**Figure 1:** Axial images of the CT scan of the orbit highlight the presence of an elliptical subperiosteal collection adjacent to the ethmoid sinuses on the left side (arrow in A). Additionally, notable soft-tissue thickening (arrowhead in B) is observed in the pre-septal region. These findings are indicative of left orbital cellulitis with a concomitant subperiosteal abscess. CT, computed tomography.

The differential diagnosis considered in this case included orbital cellulitis, pre-septal cellulitis, acute dacryocystitis, and COVID-19 infection. However, the patient's marked erythema, chemosis, tenderness to palpation, and imaging findings of subperiosteal involvement and ethmoid sinus opacification were highly suggestive of a combined pre-septal and post-septal cellulitis associated with acute dacryocystitis. The positive SARS-CoV-2 reverse transcription-polymerase chain reaction test confirmed the coexistence of COVID-19 infection.

Upon establishing the diagnosis, the patient was admitted to the pediatric ward and initiated on intravenous broad-spectrum antibiotics, including ceftriaxone and metronidazole, to cover potential pathogens, including *Staphylococcus aureus*, *Streptococcus pneumoniae*, anaerobes, and those associated with sinusitis. He was also started on oral acetaminophen for fever control.

The hospital course was characterized by a gradual improvement in periorbital swelling and erythema over the course of five days. The patient's fever subsided within 48 hours of antibiotic initiation, and there was no progression of ocular symptoms. Repeat laboratory investigations demonstrated a decreasing trend in inflammatory markers, with a C-reactive protein level of 3.2 mg/dL at the time of discharge.

Upon clinical improvement, the patient was transitioned to oral antibiotics (amoxicillin-clavulanate) for a total course of 10 days. He was discharged with instructions for close outpatient follow-up with the pediatric ophthalmology and infectious disease teams. At the follow-up visit two weeks later, the child's periorbital swelling had completely resolved, and lacrimal duct probing was scheduled to address the underlying nasolacrimal duct obstruction.

## Discussion

The presented case of a five-year-old boy with acute dacryocystitis complicated by orbital cellulitis, subperiosteal cellulitis, and ethmoid sinusitis, all occurring concurrently with COVID-19 infection, highlights several key clinical and pathophysiological aspects that warrant discussion.

Acute dacryocystitis in the pediatric population is relatively rare compared to adults [1]. Typically, it predominantly affects individuals in their 30s to 50s. However, this case emphasizes that this condition can indeed manifest in children, underscoring the importance of considering it in the differential diagnosis when faced with periorbital symptoms in pediatric patients [1]. Furthermore, the presence of subperiosteal cellulitis and ethmoid sinusitis in our patient is an unusual occurrence, adding complexity to the clinical presentation.

RETRACTED

The concomitant diagnosis of COVID-19 in our patient raises intriguing questions about the potential link between this viral infection and orbital cellulitis. While COVID-19 primarily manifests as a respiratory illness, reports of ocular symptoms and complications have emerged [2]. The exact pathogenesis of how COVID-19 may contribute to orbital cellulitis remains unclear but warrants further investigation [2,3]. It is conceivable that COVID-19-related immunomodulation and inflammation may create a favorable environment for secondary infections such as those seen in our case [2].

The diagnostic workup in our case included a contrast-enhanced CT scan, which not only confirmed the presence of acute dacryocystitis but also revealed subperiosteal cellulitis and ethmoid sinusitis [4]. These imaging findings were crucial in characterizing the extent of orbital involvement and guiding appropriate management. Furthermore, the discussion of imaging modalities, such as CT and dacryocystogram, serves to emphasize the importance of radiological evaluation in cases of orbital and lacrimal system pathology [1].

The successful management of this complex case underscores the importance of a multidisciplinary approach. Prompt initiation of broad-spectrum antibiotics, including coverage for common pathogens, was crucial in controlling the infection [5,6]. Additionally, the conservative management of the underlying nasolacrimal duct obstruction in children, as opposed to more aggressive interventions, aligns with current guidelines [5]. However, the discussion of various treatment modalities, including lacrimal probing, stenting, balloon dacryoplasty, and dacryocystorhinostomy, provides valuable insights into the spectrum of interventions available for these conditions [5].

## Conclusions

This case of a five-year-old boy with acute dacryocystitis complicated by orbital cellulitis, subperiosteal cellulitis, and ethmoid sinus opacification, concomitant with COVID-19 infection, highlights the significance of maintaining a high index of suspicion for uncommon presentations in pediatric patients, even during the ongoing pandemic. The successful management, involving prompt antibiotic therapy and conservative treatment of the underlying nasolacrimal duct obstruction, underscores the importance of a multidisciplinary approach involving pediatric ophthalmology, infectious disease, and pulmonology. The association between COVID-19 and orbital cellulitis, while intriguing, calls for further investigation. In the era of COVID-19, clinicians should remain vigilant, consider atypical manifestations, and adopt a holistic approach to the management of complex orbital and lacrimal pathologies, ensuring timely intervention for optimal patient outcomes.
